The article "Effect of Rat Medicated Serum Containing Zuo Gui Wan and/or You Gui Wan on the Differentiation of Stem Cells Derived from Human First Trimester Umbilical Cord into Oocyte-Like Cells In Vitro" was retracted in 2020. Reasons: manipulated images; duplicated images; original data or images not available.

# Effect of Rat Medicated Serum Containing Zuo Gui Wan and/or You Gui Wan on the Differentiation of Stem Cells Derived from Human First Trimester Umbilical Cord into Oocyte-Like Cells *In Vitro*

**DOI:** 10.1155/2015/825805

**Published:** 2015-01-22

**Authors:** Xiang Hu, Hua Lu, Yan-li Deng, Qian Wan, Shang-mian Yie

**Affiliations:** Department of Gynecology and Obstetrics, The Second Medical College/Teaching Hospital of Chengdu University of Traditional Chinese Medicine, Remin Nanlu Road, Chengdu, Sichuan 610041, China

## Abstract

Zuo Gui Wan (ZGW) and You Gui Wan (YGW) are two classic formulas used in clinical treatment of infertility in traditional Chinese medicine (TCM). However, the actions of the formulas remain to be proven at the cellular and molecular levels. In this study, we investigate whether the two formulas have any effect on germ cell formation and differentiation by culturing rat medicated serums containing YGW or ZGW with stem cells derived from human first trimester umbilical cord. Our results showed that while the normal rat serums had no significant effects, the rat medicated serums had significant effects on the differentiation of the stem cells into oocyte-like cells (OLCs) based on (1) cell morphological changes that resembled purative cumulus-oocyte complexes (COCs); (2) expressions of specific markers that were indicative of germ cell formation and oocyte development; and (3) estradiol production by the COC-like cells. Furthermore, ZGW medicated serums exhibited more obvious effects on specific gene expressions of germ cells, whereas YGW medicated serums showed stronger effects on estradiol production. Accordingly, our study provides evidence demonstrating for the first time that one of molecular and cellular actions of YGW or ZGW in treating human reproductive dysfunctions may be through an enhancement of neooogenesis.

## 1. Introduction

It is well known that TCM therapies were successfully used in reproductive medicine over thousands of years in China. Major theories of TCM including theories of Yin-Yang, Five Elements, Qi and Blood, and Zang-fu organs are completely different from Western medicine [1, 2]. For example, the “Kidney,” as one of the Zang-fu organs, has the ability to store congenital essence from one's parents, as well as the ability to control reproduction, growth, menstruation, conception, and aging in women [3].

Moreover, according to TCM theories, disease is generally viewed as a result of disharmony or imbalance between two opposite yet complementary forces: Yin and Yang [4]. As such, a “Kidney” Yin or Yang deficiency is the root of many reproductive disorders in both males and females. Thus, a major purpose of TCM therapies is to reinforce the Yin or Yang deficiency [4, 5].

There are a number of herbal formulas that have been successfully used to reinforce the “Kidney” Yin or Yang deficiency. Of these, ZGW and YGW are two classic formulas that have been successfully used in the clinical treatment of infertility. ZGW is usually prescribed for female patients with infertility when fertility issues arise that show signs of “Kidney” Yin deficiency. On the other hand, YGW is widely used as an herbal remedy for impotence and male infertility. For example, it has been reported that ZGW could restore ovarian functions effectively and promptly in patients with premature ovarian failure (POF) after 8 months of failed treatment with clomiphene citrate [6]. It has also been reported that YGW was useful in improving all sperm parameters, as well as facilitating the metabolism of toxins and improving general immune status [7]. Despite these studies, the actions of the two formulas remain to be proven at the cellular and molecular levels.

Germ cells are biological cells that can differentiate into mature gametes, either as eggs or sperm, of an organism that reproduces sexually. From this point of view, germ cells may correspond to the congenital essence found in TCM theories [8], and the actions of herbal formulas that reinforce the Ying or Yang deficiency may be presumed to influence germ cell fertilization abilities as well as the formation and/or differentiation of germ cells. This hypothesis has been supported by our recent studies which demonstrate that YGW decoctions can enhance the fertilizing abilities of mouse sperm* in vivo* and* in vitro* [9] and that rat medicated serums containing YGW can increase mouse oocytes* in vitro* maturation and subsequent* in vitro* fertilization abilities [10].

Stem cells are undifferentiated biological cells that can differentiate into specialized cells and can self-renew to produce more stem cells. Interestingly, a number of studies published in the past decade indicate that stem cells derived from different sources are able to differentiate into germ cells* in vitro* [11–14]. Thus, the generation of germ cells from embryonic or somatic stem cells* in vitro* may provide a valuable model for identifying factors involved in germ cell formation and differentiation.

In one of our recent reports, we demonstrated that stem cells derived from human first trimester umbilical cord (hFTUC) have an intrinsic ability to differentiate into oocyte-like cells (OLCs)* in vitro* by culturing the cells with human follicular fluid (hFF), FSH/LH, and estradiol [15]. This method provides a novel model for studying the effects of Chinese herbal medicine on the process of germ cell formation and oocyte differentiation. Accordingly, in the present study, we investigate whether or not ZGW or YGW has any effect on germ cell formation and differentiation by using this novel model that we developed.

In addition, it has been reported that serum pharmacology is more scientific and more befitting to use in TCM research than traditional pharmacology [16, 17]. In traditional pharmacology, crude drugs are directly added into a culture system of cells or organs* in vitro*. By contrast, in serum pharmacology, drugs or drug compounds are first administered to animals orally. After a period of time, the blood of the animals is then collected to separate the serum. The end result is a medicated serum that has undergone a series of biotransformation after digestion and absorption in the gastrointestinal tract. Subsequently, the medicated serum is added into a culture system of cells or organs* in vitro*. This approach is much more similar to the way in which drugs work* in vivo* [18].

Accordingly, in the present study, we first cultured hFTUC-derived stem cells in the presence of rat medicated serums containing YGW or ZGW or common herbal ingredients of the two formulas. We then compared the rat medicated serums to normal rat serums based on cell morphological changes, gene expressions indicative of germ cell formation and oocyte development, and estradiol production.

## 2. Materials and Methods

### 2.1. Isolation and Culture of hFTUC-Derived Stem Cells

Isolation and expansion of hFTUC-derived stem cells were based on a method used in our recent reports [15, 19]. Briefly, first trimester umbilical cords were collected following therapeutic pregnancy interruptions that were conducted with the written informed consent of the patients and approval from the Second Medical College/Teaching Hospital Institutional Review Board (see Supplementary Materials 1–3 available online at http://dx.doi.org/10.1155/2014/825805). The cords were rinsed several times with sterile saline and cut into pieces followed by an immersion in a 1% collagenase type I (Sigma-Aldrich, St. Louis, USA) solution for 1 hour at 37°C to isolate the stem cells. The denuded tissues were discarded after removal of the cells during digestion. The cells were pelleted by a low-speed centrifugation (250 g for 5 min) and suspended in a fresh medium. Next, the cells were plated onto a 25 cm culture flask with an expansion medium (Minimum Essential Medium Eagle, Alpha Modification; *α*-MEM, Sigma-Aldrich), which was supplemented with a 10% fetal bovine serum (Gibco-BRL, Gaithersburg, USA), 2 mmol/L L-glutamine, 50 IU/mL penicillin, and 50 mg/mL streptomycin (Gibco-BRL) in 5% CO_2_ at 37°C. The culture medium was replaced every 3 days. Subconfluent (70%–80%) cells were detached with 0.05% trypsin-0.01% EDTA (Gibco-BRL) and plated at a density of 2.4 × 10^3^ cells/cm².

### 2.2. Preparation of Rat Medicated Serums

The Animal Care and Use Committee at the Chengdu University of Chinese Traditional Medicine approved this study and all procedures as protocol number 30472225.

Three herbal decoctions were prepared by using standard methods [20]. Of the three decoctions, one decoction included YGW ingredients such as* Radix rehmanniae preparata*,* Eucommia ulmoides*,* Radix angelicae sinensis*,* Cinnamomum*,* Radix aconite lateralis preparata*,* Colla cornus cervi, Rhizoma dioscoreae*,* Fructus corni officinalis*,* Cuscuta chinensis lam*, and* Fructus lycii* and another decoction included ZGW such as* Radix rehmanniae preparata*,* Fructus corni officinalis*,* Rhizoma dioscoreae*,* Fructus lycii*,* Radix cyathulae*,* Cuscuta chinensis lam*,* Colla cornus cervi*, and* Colla carapacis et plastri testudinis*, while the third decoction included common ingredients found in ZGW and YGW (e.g.,* Radix rehmanniae preparata, Fructus corni officinalis, Rhizoma dioscoreae, Fructus lycii, Colla cornus cervi, *and* Cuscuta chinensis lam*). The three decoctions were diluted with saline (preparation : saline, 1 : 1 v/v) and stored at 4°C prior to use.

Rat medicated serums were prepared according to published protocols [21, 22]. Briefly, 160 Sprague Dawley (SD) female rats, aged 6–8 weeks and weighing 220–250 grams, were supplied by the Laboratory Animal Service Center of the Sichuan Academy of Medical Sciences and maintained in an air-conditioned room with a controlled temperature of 22 ± 2°C and a humidity level of 45–65% in a 12/12 hour light/dark cycle. The rats were randomly divided into four groups (40 in each group). The first, second, and third groups were orally administered with decoctions of YGW, ZGW, and common ingredients of ZGW/YGW, respectively. The dosage of the medicated decoctions was 20 mL/kg body weight, which was equal to 5.0 grams of formula per kg body weight. The forth group was administered with normal saline (NS) with the same volume as the medicated decoctions. Before the preparation of the serums, the rats were fasted for 16 hours and then singly administrated with either the medicated decoctions or the NS for 5 days. One hour after the last administration, blood from the rats was collected and centrifuged (3000 g for 10 min) to obtain the serums. Finally, the serums were sterilized by filtration and stored at −20°C prior to use.

### 2.3. Rat Plasma Samples Preparation for HPLC Analysis

The rat medicated serums and the normal rat serums were subjected to a high-performance liquid chromatography (HPLC) analysis by using a Shimadzu LC2010C HPLC gradient system. To perform the analysis, 1 mL of each of the serums was mixed with 5 mL of methanol and ultrasonicated for 20 min. The mixture was centrifuged at 3000 rpm for 10 min at room temperature, and the obtained supernatant was evaporated to dryness* in vacuo*. The residue was then reconstituted in 500 *μ*L of methanol solution and filtrated through a 0.45 *μ*m membrane filter (Millipore, Tokyo, Japan). Aliquots (20 *μ*L) of the filtered solution were used in the HPLC analysis.

### 2.4. Immunofluorescent Staining

Cell culturewares, which were treated for 24 days with the rat medicated serums or the normal rat serums, were washed with PBS and fixed with 4% ice-cold paraformaldehyde for 10 min. After three washes with PBS, the fixed cells were incubated for 1 hour at room temperature with one of the primary antibodies in an antibody dilution solution (Dako, Denmark). Antibodies against SP1 (1 : 100 dilution), SCP3 (1 : 100 dilution), GDF9 (1 : 100 dilution), and ZP1 or ZP2 (1 : 200 dilution) were obtained from either Santa Cruz Biotechnology (USA) or Abcam (UK). Subsequently, the cells were incubated with FITC-conjugated goat anti-rabbit antibodies (Molecular Probes) diluted at 1 : 1000 in PBS-3% (w/v) BSA for 1 hour at room temperature. After further three washes with PBS, nuclei were stained with DAPI and visualized with a fluorescence microscope.

Mouse oocytes, which had matured by the treatment of pregnant mare serum gonadotrophin (PMSG), were used as positive controls. Negative controls for immunostaining were prepared by the omission of the primary antibodies.

### 2.5. Real-Time RT-PCR Analysis

To assess the mRNA expressions of Oct4, Blimp1, Prdm14, Tfap2c, SSEA1, Stella, SCP3, GDF-9, ZP-1, ZP-2, and ZP-3, real time RT-PCR (qRT-PCR) was used as previously reported [23]. Briefly, total RNA was extracted using Trizol reagents (Invitrogen Life Technologies, Carlsbad, USA), and complementary DNA was prepared from the total RNA using oligo primers and Moloney murine leukemia virus reverse transcriptase (Applied Biosystems, Foster City, USA). qRT-PCR was then performed with the SYBR-Green mix (Applied Biosystems) on an ABI Prism 7900 sequence detector (Invitrogen). Specific primers for Oct4, Blimp1, Prdm14, Tfap2c, SSEA1, Stella, SCP3, GDF-9, ZP-1, ZP-2, ZP-3, and glyceraldehyde-3-phosphate dehydrogenase (GAPDH) are listed in Supplemental Material 5. For each PCR product, the melting curve was determined by using the comparative threshold cycle number (2^−ΔΔCt^) method, with the results being presented as fold changes in the expression of genes relative to cells cultured without the rat serums [24]. All experiments were performed in triplicate and repeated at least three times on different occasions.

### 2.6. Western Blot Analysis

To examine protein expression, cells were collected with 200 *μ*L cell lysis buffer (50 mM Tris-HCl, pH 7.4, 150 mM NaCl, 1 mM PMSF, 1 mM EDTA, 1% Triton X-100, and 1% SDS). An equal protein concentration of cell lysates per lane (10 *μ*g/lane) was separated using 10% SDS-PAGE and electroblotted to polyvinylidene fluoride (PVFD) membranes (Invitrogen, Carlsbad, CA). The membranes were blocked in PBS containing 0.05% Tween-20 (PBS-Tween) and 5% skim milk for 2 hours at room temperature and then incubated with polyclonal rabbit anti-human OCT4, Stella, GDF9, ZP1, and anti-beta-actin (Abcom UK; 1 : 500 to 1 : 1000) overnight at 4°C. Membranes were washed three times (10 min/wash) with PBS-Tween and incubated with a horseradish peroxidase-conjugated goat anti-rabbit antibody (Sigma; 1 : 2000) for 1 hr at room temperature. Membranes were washed three times again and antigen-antibody complexes were visualized with tetramethylbenzidine (TMB) (Sigma).

### 2.7. Culture Supernatant Estradiol ELISA

Estradiol concentrations in the culture supernatant were determined by an enzyme immunoassay test kit (Alpha Diagnostic International, San Antonio, USA). The assays were performed according to the manufacturer's protocol. The intra- and interassay variations were 3.5% and 10.1%, respectively. ELISAs were performed in a blinded fashion and all experiments were performed in triplicate and repeated at least three times on different occasions.

### 2.8. Data Analysis

Statistical analysis was performed using the SPSS software package (SPSS Inc., Chicago, USA). Because the data did not violate assumptions of homogeneity of variance and normal distribution, the one-way analysis of variance was used to compare the differences in the 2^−ΔΔCt^ and medium estradiol concentrations among different days of the culture and among the different experimental groups. If significance was found in the one-way analysis of variance, the data underwent post hoc comparisons. *P* < 0.05 was considered to indicate a statistically significant difference.

## 3. Results

### 3.1. Treatment of hFTUC-Derived Stem Cells with the Rat Medicated Serums or Normal Rat Serums

To test the effects of the rat medicated serums on the differentiation of hFTUC-derived stem cells into OLCs, the hFTUC-derived stem cells were cultured with *α*-MEM medium containing 2% rat medicated serums (containing either ZGW or YGW or common ingredients of ZGW/YGW). Cells cultured with normal rat serums were used as controls. In these experiments, a stem cell line in the third to fourth passages was used based on our recent report [15], which showed that cells in the third to fourth passages had the highest efficacy in the differentiation into OLCs.

Additionally, in preliminary experiments, we tested hFTUC-derived stem cells from different patients as well as the cell karyotypes of the hFTUC-derived stem cells by using an AneuVysion Multicolor DNA Probe Kit (Abbott Molecular, USA) (Supplemental Material 4). In these preliminary experiments, we did not find any significant difference in the efficiency of induction of the stem cells into the germ cell-like cells among either the cells coming from different patients or among female and male umbilical cells (average number of generation of COC-like structures or OLCs were 3–5 per 10^3^ cells). Our results here are similar to a recently published report on the effect of gender on the differentiation of mesenchymal stem cells (MSCs) into germ cells [25]. However, in order to avoid any confusion regarding the variations among the experimental groups that may be caused by cells coming from different patients or from different gender, we used a cell line with an XY karyotype in our actual experiments.

The cultures were replaced with fresh medium every 3 days and maintained for a total of 24 days. During this period, the cells changed their morphology and gradually differentiated into OLCs. Morphology of the cells was examined by using an inverted microscope (Leika DMI 3000B, Leika, Wetzlar Germany) before the medium changes. At the end of differentiation, the OLCs were examined by using immunofluorescent staining to identify whether the OLCs expressed oocyte specific markers. Meanwhile, the cells were subjected to real-time RT-PCR analysis as well as Western blot analysis at various time points to investigate gene expressions related to germ cell formation and oocyte differentiation. Further, supernatant fractions were collected from the cell cultures to determine estradiol production.

### 3.2. Effect of Rat Medicated Serum Containing Common Ingredients of ZGW/YGW on the Differentiation of hFTUC-Derived Stem Cells into OLCs

Figure 1(a) shows a representative HPLC profile for the rat medicated serum containing common ingredients of ZGW/YGW. Five distinct peaks at 2.2, 3.2, 10.8, 15.9, and 16.4 min retention times were detected in the rat medicated serum but not in the normal rat serum (Figure 1(d)).

Figure 2(a) shows that the stem cells grew adherent, exhibited spindle-like shapes, and resembled the morphologic features of undifferentiated fibroblast-like cells before the addition of the rat medicated serum. However, after 7 days of culture with 2% of the rat medicated serum, some subpopulations of the cells became morphologically distinct from the starting adherent growing cultures. From 14 to 24 days of the culture, OLCs gradually developed in a manner that was similar to what was seen previously [26] and was surrounded by smaller cells over time which resembled COCs. Occasionally, some of the OLCs reached >100 *μ*m in diameter.

To characterize the OLCs, oocyte specific markers in these cells were tested by using immunofluorescent staining on day 24 of the culture.  Figure 3(a) shows that the OLCs expressed oocyte specific markers such as SP1, SCP3, GDF9, and ZP1. Notably, the zona pellucida-like structure surrounding the OLCs could be detected in some of the cells by using anti-ZP antibodies, which was very similar to what was described in a recent report [27].

A real-time RT-PCR was performed to further verify whether the differentiated cells can be identified based on morphological changes that expressed specific gene markers related to primordial germ cells (PGC) transition and oocyte development. In the real-time RT-PCR analysis, the specificity of each amplified product in the control and differentiated cells was verified by a bidirectional sequence analysis (Supplemental Material 6). Once the specificity of the products was established, temporal changes in relative mRNA levels for each of the markers were evaluated by using GAPDH as an inner control. The Ct values for all products were below 35 and the efficiencies of targets and reference were approximately equal.

Transcripts of all the markers could be detected in the differentiated cells as well as the undifferentiated cells. However, fold changes of the differentiated versus undifferentiated cells for all the markers showed certain dynamic changes during the differentiation process. On day 7 of the differentiation, Oct4, SSEA1, and Blimp1 mRNA levels decreased by 20% and 31%, respectively, while mRNA levels of Prdm14, Tfap2c, SSEA1, and Stella increased by approximately 4.8-fold, 5.1-fold, 1.2-fold, and 9.3-fold, respectively (*P* = 0.037, 0.035, 0.118, and 0.001, resp.) when compared to levels obtained on day 0 (Figure 4(a)). On day 24 of the differentiation, in which OLCs developed, the mRNA levels of SCP3, GDF9, ZP1, and ZP2 increased by approximately 1.4-fold (*P* = 0.004), 4.8-fold (*P* = 0.033), 6.7-fold (*P* = 0.031), and 2.2-fold (*P* = 0.046), respectively, while the mRNA levels in ZP3 showed no changes when compared to levels obtained on day 0 (Figure 4(a)).

In the western blot analysis, protein expressions of Stella on day 7 and GDF-9 and ZP1 on day 24 after the treatment were obviously increased while Oct4 protein expression had a slight decrease from day 0 to day 24 (Figure 5(a)). These changes in protein expressions were similar to those of the mRNA expressions.

Estradiol concentrations in the cultured medium on day 0 was 3.7 ± 0.18 pg/mL with the levels of estradiol in cultured medium gradually increasing from 14.6 ± 0.23 to 26.0 ± 0.30 pg/mL during days 15 to 21 of the treatment (*F* = 39.3, *P* = 0.0001; Figure 6(a)).

### 3.3. Effect of Rat Medicated Serum Containing YGW on the Differentiation of hFTUC-Derived Stem Cells into OLCs

Figure 1(b) shows a representative HPLC profile for the rat medicated serum containing YGW. Seven distinct peaks at 3.5, 3.8, 8.8, 12.3, 16.7, 17.2, and 21.6 min retention times were detected in the rat medicated serum but not in the normal rat serum (Figure 1(d)).

Similar to the rat medicated serum containing common ingredients of YGW/ZGW, Figure 2(b) shows that some subpopulations of the cells became morphologically distinct from the starting cultures after 7 days of culture with 2% of the rat medicated serum containing YGW. On day 24 of the differentiation, OLCs surrounded by smaller cells also appeared.

Figure 3(b) shows that the OLCs expressed SP1, SCP3, GDF9, and ZP1 as detected by using immunofluorescent staining. In the real-time RT-PCR analysis, fold changes of differentiated versus undifferentiated cells for all of the markers showed certain dynamic changes during the differentiation process. On day 7 of the differentiation, Blimp1 mRNA levels decreased by 75% (*P* = 0.005) and SSEA1 mRNA levels remained unchanged (96%), while mRNA levels of Oct4, Prdm14, Tfap2c, and Stella increased by approximately 1.38-fold, 10.16-fold, 4.97-fold, and 8.1-fold, respectively (*P* = 0.114, 0.02, 0.009, and 0.001, resp.) when compared to levels obtained on day 0 (Figure 4(b)). On day 24 of the differentiation, in which OLCs developed, the mRNA levels of SCP3, GDF9, ZP1, and ZP3 increased by approximately 1.62-fold (*P* = 0.018), 6.05-fold (*P* = 0.043), 27.9-fold (*P* = 0.036), and 2.49-fold (*P* = 0.048), respectively, while the mRNA levels of ZP3 decreased by 51% (*P* = 0.035) when compared to levels obtained on day 0 (Figure 4(b)).  Figure 5(b) showed that protein expressions of Stella on day 7, GDF-9 on day 24, and ZP1 on day 7 and day 24 after the differentiated were increased while no clear changes in Oct4 protein expression during the differentiation were observed.

Estradiol concentrations in the cultured medium on day 0 was 6.0 ± 0.60 pg/mL with the levels of estradiol in cultured medium gradually increasing and reaching 28.3 ± 1.41 pg/mL by day 9, which remained at this high level until day 21 of the treatment (*F* = 62.6, *P* = 0.0001; Figure 6(b)).

### 3.4. Effect of Rat Medicated Serum Containing ZGW on the Differentiation of hFTUC-Derived Stem Cells into OLCs

Figure 1(c) shows a representative HPLC profile for the rat medicated serum containing ZGW. Six distinct peaks at 2.2, 3.2, 11.3, 16.6, 17.0, and 22.6 min retention times were detected in the rat medicated serum but not in the normal rat serum (Figure 1(d)).

Similar to rat medicated serums containing common ingredients of YGW/ZGW and YGW, after 7 days of culture with 2% of the rat medicated serum containing ZGW, some subpopulations of the cells also became morphologically distinct from the starting cultures, and OLCs developed from days 14 to 24 (Figure 2(c)).

The OLCs expressed proteins of SP1, SCP3, GDF9, and ZP1 as detected by immunofluorescent staining (Figure 3(c)). The expressions of levels of mRNA in Oct4, Blimp1, Prdm14, Tfap2c, SSEA1, and Stella increased by approximately 3.77-fold (*P* = 0.009), 1.42-fold (*P* = 0.027), 2.80-fold (*P* = 0.006), 14.1-fold (*P* = 0.001), 1.17-fold (*P* = 0.165), and 36.7-fold (*P* = 0.001) on day 7 when compared to levels obtained on day 0 (Figure 4(c)). Meanwhile, after 24 days, the mRNA levels of SCP3, GDF9, ZP1, ZP2, and ZP3 increased by approximately 2.8-fold (*P* = 0.019), 15.5-fold (*P* = 0.016), 2.7-fold (*P* = 0.018), 3.89-fold (*P* = 0.01), and 1.88-fold (*P* = 0.007) when compared to levels obtained on day 0 (Figure 4(c)). Similarly, the western blot analysis showed that the protein expressions of OCT4 and Stella on day 7 and GDF-9 and ZP1 on day 24 after treatment were obviously increased (Figure 5(c)).

Estradiol concentrations in the cultured medium on day 0 were 4.0 ± 0.2 pg/mL with the levels of estradiol in cultured medium gradually increasing and reaching a peak value of 30.0 ± 1.52 pg/mL by day 9. Afterward, the estradiol levels decreased but were still higher than day 0 until day 21 of the treatment (*F* = 36.0, *P* = 0.0001; Figure 6(c)).

### 3.5. Effect of Normal Rat Serum on the Differentiation of hFTUC-Derived Stem Cells

Normal rat serum was used as a control to demonstrate the effects of the rat medicated serums on the differentiation of hFTUC-derived stem cell into OLCs. Figure 1(d) shows a representative HPLC profile for the normal rat serum. Only one peak at 2.75 min retention times was detected.

During the 24 days of culture with 2% of the normal rat serum, the morphology of cells remained the same as the morphologic features of undifferentiated fibroblast-like cells (Figure 2(d)). Immunofluorescent staining showed no positive reaction with anti-SP1, -SCP3, -GDF9, and -ZP1 antibodies in during the 24 days of culture (Figure 3(d)). In the real-time RT-PCR analysis, there were no significant fold changes in the mRNA levels of Oct4, Blimp1, Tfap2c, SSEA1, and Stella while the mRNA level of Prdm14 increased by 1.3-fold (*P* = 0.045) after 7 days when compared to levels obtained on day 0 (Figure 4(d)). On day 24, there were no significant changes in the mRNA levels of SCP3 and GDF9, while the mRNA levels of ZP1 and ZP3 decreased by 85% (*P* = 0.01) and 70% (*P* = 0.02), respectively, when compared to levels obtained on day 0 (Figure 4(d)). The unchanged mRNA levels of Oct4, Stella, GDF9, and ZP1 were also confirmed by their protein expression assayed with the western blotting (Figure 5(d)).

Estradiol concentrations in the cultured medium on day 0 was 3.8 ± 0.20 pg/mL with the levels of estradiol in cultured medium increasing slightly to 8.42 ± 0.42 and 7.6 + 0.39 pg/mL by days 12 and 15 of the treatment, respectively (*F* = 2.15, *P* = 0.096; Figure 6(d)).

### 3.6. Comparison of the Effect of the Three Types of Rat Medicated Serums on Gene Expressions Related to Germ Cell Formation, Oocyte Development, and Estradiol Production

Although the three types of rat medicated serums contained different active herbal ingredients and/or biotransformed components based on the HPLC analysis, no significant differences in cell morphologic changes and protein expressions of oocyte markers, such as SP1, SCP3, GDF9, and ZP1, were observed among the rat medicated serums. However, the effects of the three types of rat medicated serums on gene transcripts related to germ cell formation and oocyte development as well as estradiol production were observed to be different. In particular, as shown in Figure 7, mRNA levels of Oct4, Blimp1, Prdm14, Tfap2c, and Stella in the rat medicated serum containing ZGW were significantly higher than those in the other two types of rat medicated serums after 7 days of treatment. The mRNA levels of SCP3 and GDF-9 in the rat medicated serum containing ZGW were also significantly higher than those in the other two types of rat medicated serums after 24 days of treatment. However, no significant differences in the mRNA levels of SSEA1, ZP-1, ZP-2, and ZP-3 were detected among the rat medicated serums. Interestingly, COC-like cells induced by the rat medicated serum containing YGW produced more estradiol when compared to the rat medicated serum containing ZGW or the rat medicated serum containing common herbal ingredients of ZGW/YGW (*P* = 0.042 and 0.048, resp., Table 1). Note that no significant difference was found in the average numbers of OLCs among the three treatment groups (4.0 ± 0.36 versus 3.8 ± 0.40 versus 4.1 ± 0.40 (mean ± SE) for common herbal ingredients of ZGW/YGW versus YGW versus ZGW). Accordingly, the differences in the estradiol production could be attributed to the different effects of the three types of medicated serums.

## 4. Discussion

Many studies have shown that OLCs can be generated from embryonic stem cells (ESCs), induced from pluripotent stem cells (iPSc) and adult stem cells* in vitro* [11, 26–32]. In these previous studies, the induction of ESCs or somatic stem cells into OLCs was generally performed by culturing the cells with growth factors [28, 30], estrogenic stimuli [12], conditional medium from testicular cell cultures [33], follicular fluid, and gonadotrophins [15, 26, 27] or with ovarian granulose cells [29]. In the present study, we showed that hFTUC-derived stem cells are also able to differentiate into OLCs by the treatment of rat medicated serums containing ZGW or YGW or common ingredients of ZGW/YGW. The germ cell precursors in our study showed close resemblance to oocytes, which were based on (1) morphologic changes; (2) marker expression profiles at the mRNA and/or protein levels; and (3) production of estradiol from COC-like structures. By contrast, no significant morphological changes, germ cell marker expressions, or estradiol productions were found in the cells treated with normal rat serum.

Germ cell development requires a series of multiple well-orchestrated steps, which involve the concurrent up- and downregulation of specific determinant gene expressions [34]. It has been demonstrated that Blimp1, Prdm14, and Tfap2c are key germ cell determinants for regulating PGC specification [35], and Oct4 is proposed to be required for the survival of primordial germ cells [36]. In the present study, the rat medicated serums caused an increase in the mRNA levels of Oct4, Blimp1, Prdm14, and Tfap2c after 7 days of treatment, although the effects were different among the rat medicated serums.

Moreover, the PGC-like cells also expressed SSEA1 and Stella, which are markers indicative of germ cell formation. It has been reported that human germ cells express SSEA1 [37], and Stella plays a role in facilitating germline and endodermal differentiation of human ES cells [38]. A lack of Stella expression at an earlier stage could indicate a transition of cells into the germ lineage [33].

Further, the rat medicated serums caused an increase in the levels of mRNA of oocyte specific markers such as SP1, SCP3, GDF-9, ZP1, ZP2, and ZP3 during the differentiation process. SCP3 is a meiosis-specific protein [39], while GDF-9 is required for normal folliculogenesis [40], and zona pellucida glycoproteins are expressed only in oocytes [41]. The SP1 protein, which could promote rapid germ-cell differentiation [42], was also detected in the COC-like cells/OLCs. Accordingly, our results indicate that the rat medicated serums have the potential to induce the differentiation of hFTUC-derived stem cells into OLCs.

Moreover, the detection of estradiol production in our cultures provides evidence for the functional activity of somatic cells around the OLCs, since the 4–8-fold increase in estradiol concentrations over the controls on day 21 should be due to the COC-like cells. However, further investigation is needed to confirm the existence and function of granulosa cell-like cells in the COC-like cells.

The HPLC profiles revealed that the rat medicated serum containing ZGW had six distinct peaks (at 2.2, 3.2, 11.3, 16.6, 17.0, and 22.6 min retention times), the rat medicated serum containing YGW had seven distinct peaks (at 3.5, 3.8, 8.8, 12.3, 16.7, 17.2, and 21.6 min retention times), and the rat medicated serum containing common ingredients of ZGW/YGW had five distinct peaks (at 2.2, 3.2, 10.8, 15.9, and 16.4 min retention times). At least 3 peaks, at 2.2, 3.2, and 16 min retention times, were similar in all three types of rat medicated serums. Since the three types of rat medicated serums have similar effects on the differentiation of OLCs, the common distinct peaks may represent active herbal ingredients and/or biotransformed components in the rat medicated serums that are responsible for the induction of cell specific differentiation in terms of cell morphological changes and expressions of SCP3, GDF9, and ZP1 or ZP2 proteins. However, the rat medicated serum containing ZGW had stronger effects on mRNA expressions of genes related to germ cell formation and oocyte development, while the rat medicated serum containing YGW showed more obvious influence on estradiol production. The findings were also confirmed by the western blot analysis since protein expressions of Oct4, Stella, GDF9, and ZP1 from day 0 to day 24 of the differentiation have a similar changing pattern to that of mRNA levels. This suggests that other distinct peaks in these two types of rat medicated serums may be responsible for the differences. Our findings are consistent with clinical observations that ZGW could restore ovarian functions effectively and promptly [5, 6, 8] and with a previous report that showed that YGW can enhance estradiol secretion by mice granulose cells* in vitro* [43].

Moreover, one of our recent studies showed that rat medicated serums containing YGW had a significant effect on mouse oocyte maturation* in vitro* via molecular signal pathways similar to those induced by FSH [10]. The results suggest that some active or biotransformed herbal ingredients in the medicated serums may have gonadotrophin functions to stimulate the production of estradiol from differentiated granulosa cells.

Following the development of tissue engineering and cell therapy, stem cell transplantations are emerging as an important research topic due to their therapeutic potentials in a variety of diseases. For example, investigations into the application of MSCs in improving liver fibrosis have been carried out in animal models and clinical trials [44]. Because stem cells are able to differentiate into germ cell-like cells* in vitro* [11–14], stem cell therapy may also become an important research topic in the future due to their therapeutic potentials in reproductive diseases such as POF. Interestingly, it has been reported that the differentiation, proliferation, and migration of MSCs can be regulated by a combination of TCM treatments [44], which may be of great benefit for infertility therapy in the future.

According to TCM theories, the “Kidney” houses the reproductive essence (jing) and governs reproduction [45]. In modern terminology, the essence refers to eggs and sperm, the most primordial building blocks of reproduction [8]. While the “Kidney” essence correlates with eggs and sperm, the “Kidney” Yin and “Kidney” Yang can be thought of as the hormonal underpinnings of the reproductive system [8]. Because YGW and ZGW are used in patterns with “Kidney” Yang and Yin deficiency, respectively, they may regulate the endocrine function to promote germ cell transition, although other important underlying mechanisms may be also involved. However, this hypothesis needs to be experimentally demonstrated in future studies by using isolated herbal ingredients. Additionally, future studies are needed to identify the chemical compositions and properties of these herbal ingredients.

## 5. Conclusion

In summary, we have demonstrated that rat medicated serums containing YGW or ZGW or common ingredients of ZGW/YGW can induce the differentiation of hFTUC-derived stem cells into OLCs* in vitro*. We also showed that the rat medicated serum containing ZGW has more obvious effects on gene transcript expressions related to germ cell transition determination and oocyte development than the other two types of rat medicated serums. Further, the rat medicated serum containing YGW showed stronger effects on estradiol production by COC-like cells. Our findings suggest that one of actions of the ZGW and YGW formulas is an enhancement of neooogenesis. This should play an important role in the understanding of the pharmacological mechanisms of ZGW or YGW at the cellular and molecular levels in treating human reproductive dysfunctions such as premature ovarian failure. Consequently, this can lead to better clinical practices in the future which combine both TCM and modern reproductive medicine. Nevertheless, further studies are necessary in order to identify which active ingredients and/or biotransformed components are responsible for the underlying mechanisms of the herbal formulas.

## Supplementary Material

Supplemental Material 1: Voluntary donation abortion organizations informed consent (Chinese Version)
Supplemental Material 2: Voluntary donation abortion organizations informed consent (English Version)
Supplemental Material 3: Ethics statement certified by the hospital ethics committee
Supplemental Material 4: Human FTUC stem cell karyotyping test and results
Supplemental Material 5: List of the primers used in the qPCR analysis
Supplemental Material 6: Report on sequence analysis from a nucleic acid sequencing service corporation

## Figures and Tables

**Figure 1:** HPLC profiles of the rat medicated serums after oral administration of the decoctions. (a) Rat medicated serum after 1 hour of oral administration of the decoction with common ingredients of ZGW/YGW; (b) rat medicated serum after 1 hour of oral administration of the decoction with YGW; (c) rat medicated serum after 1 hour of oral administration of the decoction with ZGW; and (d) normal rat serum. Several distinct peaks (red color arrows) are detected in the rat medicated serums but not in the normal rat serum. This indicates that the rat medicated serums may contain certain active ingredients and/or metabolic components.

**Figure 2:** Effect of rat medicated serums on morphological changes of inducing stem cells into oocyte-like cells. (a), (b), and (c) show representative images of stem cells treated with the rat medicated serums containing common ingredients of ZGW/YGW, YGW, and ZGW, respectively. On day 7, some subpopulations of the cells appeared to be morphologically distinct from the cells on day 0, which resembled PGC (green arrows). On day 24, OLCs developed and were surrounded by smaller cells that showed resemblance to follicular structures (red arrows). Higher magnification images of OLCs are also presented to show that they are in pachytene. (d) shows representative images of stem cells treated with normal rat serum. No significant morphological changes were found during the entire period of 24 days. Scale bar is set to 100 *μ*m.

**Figure 3:** Detection of oocyte markers in OLCs by immunofluorescent analysis. (a), (b), and (c) show immunofluorescent stains of SP1, SCP3, GDF9, and ZP1 or ZP2 in OLCs on day 24 after treatment with the rat medicated serums containing common ingredients of ZGW/YGW, YGW, and ZGW, respectively. (d) shows the immunofluorescent analysis of expressions of SP1, SCP3, GDF9, and ZP1 in stems cells treated with normal rat serum. (e) shows negative controls obtained by incubating the stems cells with secondary anti-rabbit or anti-mouse antibody alone after staining with DAPI. Scale bar is set to 50 *μ*m.

**Figure 4:** Detection of germ cell and oocyte markers in germ cell-like cells and OLCs by real-time RT-PCR. Real-time RT-PCR analysis of expressions of germ cell markers (OCT4, SSEA-1, Stella, Blimp1, Prdm14, and Tfap2c) in the PGC-like cells after 7 days of differentiation and oocyte markers (SCP3, GDF9, ZP1, ZP2, and ZP3) after 24 days of treatment with the rat medicated serums containing common ingredients of ZGW/YGW (a), YGW (b), ZGW (c), and normal rat serum (d). Relative mRNA levels are normalized for the GAPDH housekeeper. The results are presented relative to the control cells (2^−ΔΔCt^). Data represents the mean ± SEM of three independent experiments. ∗ indicates statistical significance when compared to day 0 of the culture.

**Figure 5:** Western blot analysis of protein expression. (a), (b), and (c) show western blotting of expressions of Oct4 (MW = 45 kd), Stella (MW = 23 kd), GDF9 (MW = 51 kd), and ZP1 (MW = 70 kd) on day 0, day 7, and day 24 after treatment with the rat medicated serums containing common ingredients of ZGW/YGW, YGW, and ZGW, respectively. (d) shows western blotting of expressions of Oct4, Stella, GDF9, and ZP1 in stems cells treated with normal rat serum. Beta-actin (MW = 42 kd) was used as an internal control.

**Figure 6:** Determination of changes of estradiol production. Estradiol production during the treatment with the rat medicated serums containing common ingredients of ZGW/YGW (a), YGW (b), ZGW (c), and normal rat serum (d). Data represents the mean ± SEM of three independent experiments. During 24 days of treatment, estradiol productions of OLCs were gradually increased in the three rat medicated serum groups (all *P* values = 0.0001, one-way analysis of variance) while no significant difference was detected in cultures treated with normal rat serum (*P* = 0.092). ∗ indicates statistical significance when compared to day 0 of the treatment.

**Figure 7:** Comparison of the effect of the three types of rat medicated serums on gene expressions. Significant differences in the mRNA levels of Oct4, SSEA-1, Stella, Blimp1, Prdm14, and Tfap2c can be seen on day 7, with the highest expression seen in the stem cells treated with the rat medicated serum containing ZGW. No significant difference in any of the gene expressions was found on day 24, except for Tfap2c. On day 24, the mRNA levels of SCP3 and GDF-9 in the rat medicated serum containing ZGW were higher than the mRNA levels of SCP3 and GDF-9 in the other two types of rat medicated serums. No significant differences in mRNA levels of ZP-1, ZP-2, and ZP-3 were detected among the three types of rat medicated serums.

**Table 1:** Comparison of estradiol production from the differentiated cells treated with rat medicated serums containing common components of YGW and ZGW, YGW, or ZGW.

Comparison of	*F*	*P*
NS versus YGW/ZGW	33.88	0.006
NS versus YGW	60.42	0.00035
NS versus ZGW	35.98	0.0054
YGW/ZGW versus YGW	2.47	0.042
YGW/ZGW versus ZGW	1.53	0.167
YGW versus ZGW	2.45	0.048
